The article "PD-1 Is an Immune-Inflammatory Potential Biomarker in Cerebrospinal Fluid and Serum of Intractable Epilepsy" was retracted in 2024. Reasons: signs of a paper mill; compromised peer review; unreliable results or conclusions.

# PD-1 Is an Immune-Inflammatory Potential Biomarker in Cerebrospinal Fluid and Serum of Intractable Epilepsy

**DOI:** 10.1155/2021/7973123

**Published:** 2021-03-17

**Authors:** Hong Tang, Xuefeng Wang

**Affiliations:** ^1^Department of Critical Care Medicine, The First Affiliated Hospital of Chongqing Medical University, China; ^2^Department of Surgical Intensive Care Unit, The First Affiliated Hospital of Chongqing Medical University, China; ^3^Department of Neurology, The First Affiliated Hospital of Chongqing Medical University, 1 Youyi Road, Chongqing 400016, China; ^4^Chongqing Key Laboratory of Neurology, Chongqing, China

## Abstract

**Purpose:**

Previous studies have demonstrated that immune and inflammatory factors play an important role in recurrent seizures. The PD-1-PD-L pathway plays a central and peripheral immunosuppressive role by regulating multiple signaling pathways during the inflammatory and immunologic processes. This study is aimed at assessing PD-1 levels in cerebrospinal fluid (CSF) and serum samples from patients with intractable epilepsy.

**Methods:**

PD-1 levels were assessed in CSF and serum samples from 67 patients with intractable epilepsy (41 and 26 individuals with partial seizure and intractable status epilepticus, respectively) and 25 healthy controls, using flow cytometric analysis and sandwich enzyme-linked immunosorbent assays (ELISA).

**Results:**

Serum-PD-1+CD4^+^CD25^high^ Treg levels in the experimental groups and the control group were 10.26 ± 2.53 (PS group), 35.95 ± 27.51 (ISE group), and 4.69 ± 2.44 (control group). In addition, CSF-PD-1 level in patients with epilepsy was higher than that in the control group (50.45 ± 29.56 versus 19.37 ± 4.51), indicating a statistically significant difference (*P* < 0.05). Interestingly, serum- and CSF-PD-1 levels in individuals with epilepsy were not affected by antiepileptic drug and treatment course, but by epilepsy onset level. Of note, the increase of CSF- and serum-PD-1 levels was more pronounced in subjects with intractable status epilepticus than those with partial seizure.

**Conclusion:**

Serum- and CSF-PD-1 levels constitute a potential clinical diagnostic biomarker for intractable epilepsy and could also be used for differential diagnosis.

## 1. Introduction

Epilepsy is a common, serious chronic neurological disease [1] associated with stigma, psychiatric comorbidity, and high economic costs that caused the 56.79 per 100,000 person-years of incidence rate of epilepsy and affects about 50 million people worldwide [2]. Dozens of antiepileptic drugs (AEDs) have been developed and have good efficacy on epileptic seizures; nonetheless, approximately 20%-30% of patients remain untreated and often experience side effects [3, 4]. The positive rate of electroencephalogram is very low so it is difficult to diagnose epilepsy in clinic. Many patients are misdiagnosed or missed depending only on their clinical manifestations. Therefore, in order to improve the diagnosis rate of epilepsy, we need to find a new diagnostic biomarker.

The article "PD-1 Is an Immune-Inflammatory Potential Biomarker in Cerebrospinal Fluid and Serum of Intractable Epilepsy" was retracted in 2024. Reasons: signs of a paper mill; compromised peer review; unreliable results or conclusions.

At present, the research of epilepsy mostly focuses on neurotransmission. The imbalance between excitatory and inhibitory neurotransmission and the formation of abnormal epilepsy network are accepted as the common mechanism of various epileptic seizures. With the exploration of pathogenesis of epilepsy, a large number of evidences show that recurrent seizures may be related to nonneural changes in recent years, but infections and infestations are among the most common risk factors for seizures and acquired epilepsy [5–9]. Immune and inflammatory factors play an important role in recurrent seizures [10–12]. The reported risk of unprovoked seizures in population-based cohorts of survivors with CNS infections from developed countries is between 6.8 and 8.3%, much higher than that in resource-poor countries [7]. Meanwhile, the sterile (noninfectious) inflammatory response can also occur in various brain insults in the absence of an infectious agent, which can induce the initiation of molecular mechanism and signal pathways of immune inflammation and then promote the genesis and recurrent seizures [13]. Furthermore, autoimmune encephalitis as a cause of epileptic status is also increasingly recognized as an important position [7]. Therefore, understanding the immuno-inflammation mechanisms of neurotransmission is necessary for exploring novel antiepileptic targets.

Programmed cell death protein 1 (PD-1), which was initially considered to be a molecule that regulates cell death [14], has now been identified as a key checkpoint inhibitory receptor that alters the function of T cells after antigen-mediated stimulation. The PD-1-PD-L pathway plays a central and peripheral immunosuppressive role by regulating multiple signaling pathways. PD-1 mediates the inhibitive effect of T cells by antagonizing T cell receptor-mediated signal transduction and regulating activated T cells; it maintains the inhibition of T cell response by inducing iTreg (induced Treg cells) and then plays an important inhibitory role [15–17]. Therefore, PD-1 and regulatory CD4^+^CD25^high^ T cells (Tregs) have become key players in immune regulation. There are innate immune activity and acquired adaptive immunity in the process of epilepsy [18]. In addition, immune inflammatory factors are also one of the important reasons for recurrent seizures in intractable epilepsy (IE). Considering the function of PD-1 and its possible role, we hypothesized that PD-1 may be altered in the CSF and serum concentration in intractable epilepsy. Here, PD-1 concentrations were measured in CSF and serum samples from patients with IE as well as from controls who underwent lumbar punctures as part of a medical evaluation to assess the group differences.

The article "PD-1 Is an Immune-Inflammatory Potential Biomarker in Cerebrospinal Fluid and Serum of Intractable Epilepsy" was retracted in 2024. Reasons: signs of a paper mill; compromised peer review; unreliable results or conclusions.

## 2. Patients and Methods

### 2.1. Ethics Statement

The study was performed in accordance with the Declaration of Helsinki of the World Medical Association. A written informed consent form for the use of CSF and peripheral blood in research was obtained from all patients and controls enrolled. Informed consent of critical patients with ISE is required and obtained from the legally authorized patient representatives, due to the fact that patients with ISE admitted to the ICU were judged to be too seriously ill to provide valid consent (Ethics Committee of the First Affiliated Hospital of Chongqing Medical University, Chongqing, China, ethical document no. 2020-162).

### 2.2. Patients

Subjects of intractable epilepsy with partial epilepsy (PS) were recruited from the Epilepsy Clinic. Subjects of intractable epilepsy with intractable status epilepticus (ISE) were recruited from the inpatient, Department of Neurology, The First Affiliated Hospital of Chongqing Medical University. Epilepsy was diagnosed and classified by two experts at our epilepsy center according to the criteria proposed by the International League Against Epilepsy in 2001. Patients underwent comprehensive clinical examination, including medical history, electroencephalography assessment, neurological and psychiatric examinations, and cranial magnetic resonance imaging (MRI). All examinations (neurological and psychiatric examinations and MRI) returned normal results.

Samples of peripheral blood from 67 patients with IE (32 males and 34 females) were collected. Samples of CSF from 26 patients with intractable status epilepticus (ISE) (13 males and 13 females) were collected by lumbar puncture. Patient ages ranged from 19 to 46 years. Forty-one patients had partial seizure. Twenty-six patients had generalized tonic-clonic seizure.  Table 1 summarizes the seizure types, durations, and ages of the patients assessed here. The experimental group was subdivided into two (the group with partial epilepsy (PS) and the group with intractable status epilepticus (ISE)) groups. Criteria for IE included the following: seizure events for at least 2 years, use of at least three AEDs (antiepileptic drugs), and absence of structural lesion in the brain tissue as assessed by MRI and CT; patients with NIE were those with good response to AEDs and no seizure recurrence. No patient with epilepsy enrolled in this study had a seizure within 24 h of sample collection. The control samples were obtained from 25 controls with mild dizziness and headache, no history of epilepsy or other central nervous diseases, no anxiety or depression, and not currently taking any medication. Routine clinical examination and cranial magnetic resonance imaging (MRI) did not reveal any central nervous diseases such as cerebral ischemia, hemorrhage, inflammation, and tumor. The diagnosis was carried out by two independent neurologists. Lumbar puncture was performed to further rule out central nervous system disorders.

The article "PD-1 Is an Immune-Inflammatory Potential Biomarker in Cerebrospinal Fluid and Serum of Intractable Epilepsy" was retracted in 2024. Reasons: signs of a paper mill; compromised peer review; unreliable results or conclusions.

Patient with epilepsy enrolled in this study had a seizure within 24 h of sample collection. For each subject, 2 ml of CSF and 5 ml of venous blood samples were collected in k3 EDTA vials. The flow cytometry was completed within 4 hours. The supernatant of cerebrospinal fluid and serum was stored at -80°C, and the cytokines were determined by ELISA.

### 2.3. Exclusion Criteria

The patients with pseudoseizure and secondary epilepsy; infectious diseases in the last month; and HBV, HIV, tuberculosis, syphilis, and cancer or receiving immunosuppressive therapy for other associated illness were excluded.

### 2.4. Flow Cytometric Analysis

Ficoll density gradient centrifugation method was used to separate PBMC which was then cultured in RPMI 1640 medium under the stimulation of activator. Then, trypan blue staining was used to detect and count the alive cells. The untreated cells were used as negative control. Cells were permeabilized and fixed according to the manufacturer's protocol followed by staining. The experimental groups were added anti-CD4FITC, anti-CD25-PE, and anti-PD-1-APC (BioLegend, USA) at room temperature in the dark, for 30 min at 4°C. CD4^+^ T lymphocytes were used to set the door for reading. The samples were detected and sorted by flow cytometry; more than 50,000 cells were acquired in each tube for flow cytometric analyses on BD FACSCalibur.

### 2.5. Determination of IL-10/IL-6 with ELISA Method

The IL-10/IL-6-coated antibody was diluted according to the concentration. After incubation in 37°C incubator for 90 min then washing, add biotinylated antibody working solution. After incubation in 37°C incubator then washing, add the working solution of enzyme binding compound. After incubation in 37°C incubator then washing, add developer then incubate in 37°C incubator for 10-15 min in the dark. Measure the od450nm value immediately after adding the termination solution and mixing.

### 2.6. Statistical Methods

Statistical analysis was performed with SPSS 24.0 (SPSS, USA). Data are mean ± standard deviation (SD). Differences between the groups with epilepsy and the control group were assessed by independent samples *t*-test, while nonnormal distribution of measurement data was used by chi-square test and Kruskal-Wallis rank sum test. The correlation analysis among age, gender, course of disease, and the results was calculated by Spearman correlation. *P* < 0.05 was considered statistically significant.

The article "PD-1 Is an Immune-Inflammatory Potential Biomarker in Cerebrospinal Fluid and Serum of Intractable Epilepsy" was retracted in 2024. Reasons: signs of a paper mill; compromised peer review; unreliable results or conclusions.

## 3. Result

### 3.1. Clinical Characteristics of Subjects

The clinical characteristics of subjects are shown in Table 1.

### 3.2. Compared with the Control Group, the Changes of Immune Inflammation in Peripheral Blood of Patients with Intractable Epilepsy

The total number of lymphocytes and CD4^+^ cells in the peripheral blood of patients with IE decreased. (1) The positive rate of lymphocytes in each group was as follows: control group 13.22 ± 6.41, PS group 6.63 ± 5.49, and ISE group 3.92 ± 3.32; the epilepsy groups were significantly lower than the control group; the ISE group was significantly lower than the PS group (*P* < 0.05) (Figure 1(a), Table 1.2). (2) The expression rate of CD4^+^ in each group was as follows: control group 38.64 ± 6.64, PS group 34.20 ± 8.89, and ISE group 29.87 ± 9.23; the epilepsy groups were significantly lower than the control group; the ISE group was significantly lower than the PS group (*P* < 0.05) (Figure 1(b), Table 1.2).

PD-1 was upregulated in CD4^+^CD25^high^ Treg cells, and IL-10 was upregulated simultaneously in the peripheral blood of patients with intractable epilepsy. (1) The expression rate of PD-1+CD4^+^CD25^high^ Treg in each group was as follows: control group 4.69 ± 2.44, PS group 10.26 ± 2.53, and ISE group 35.95 ± 27.51; the epilepsy groups were significantly higher than the control group; the ISE group was significantly higher than the PS group, with statistical difference (*P* < 0.05) (Figure 2(a), Table 1.2). (2) The correlation analysis of the ratio of PD-1+CD4^+^CD25^high^ Treg/CD4^+^CD25^high^ Treg for three groups of subjects and comparison between the each pair groups showed that the *Z* values were as follows: -4.654 (control and PS), -6.994 (control and ISE), and -3.364 (PS and ISE). The above ratio was significantly increased in epileptic patients and increased with the degree of attack, with statistical difference (*P* < 0.05) (Figure 2(b), Table 1.3). (3) The correlation between the results of two groups of intractable epilepsy and the age, gender, course of disease, and seizure frequency was analyzed. The correlation coefficients of the PS group were as follows: PD-1+CD4^+^CD25^high^ Treg (-0.301), PD-1+CD4^+^CD25^low^ Treg (-0.333^∗^), CD4^+^CD25^low^ (0.305), CD4^+^CD25^high^ (0.045), IL-10 (-0.247), P1 (0.081), P2 (-0.335^∗^); only the age of patients in the PS group and the percentage of PD-1+CD4^+^CD25^low^ Treg cells and the percentage of CD4^+^ T cells (P2) were correlated, and the expression decreased with the increase of age (*P* < 0.05). There was no correlation between sex, course of disease, and attack frequency and the results in the PS group. There was no statistical difference between age, sex, course of disease, and attack frequency and the results in the ISE group (Figure 2(c), Tables 1.4 and 1.5). (4) IL-10 concentration in serum was as follows: control group 54.52 ± 11.04 pg/ml, PS group 79.46 ± 18.22 pg/ml, and ISE group 220.22 ± 9.87 pg/ml; the epilepsy groups were significantly higher than the control group; the ISE group was significantly higher than the PS group; there was a statistical difference (*P* < 0.05) (Figure 2(d), Table 1.2). (5) IL-6 concentration in serum was as follows: control group 7.56 ± 3.88 pg/ml, PS group 13.18 ± 5.85 pg/ml, and ISE group 13.97 ± 4.33 pg/ml; the epilepsy groups were significantly higher than the control group (*P* < 0.05); there was no statistical difference between the ISE group and the PS group (Figure 2(e), Table 1.2).

The article "PD-1 Is an Immune-Inflammatory Potential Biomarker in Cerebrospinal Fluid and Serum of Intractable Epilepsy" was retracted in 2024. Reasons: signs of a paper mill; compromised peer review; unreliable results or conclusions.

### 3.3. Compared with the Control Group, the Changes of Immune Inflammation in Cerebrospinal Fluid of Patients with Intractable Epilepsy

The total number of lymphocytes in cerebrospinal fluid of IE increased, and there was no significant difference in the expression rate of CD4^+^. (1) The positive rate of lymphocytes in the control group (3.68 ± 4.91), the ISE group (6.05 ± 5.57), and the epilepsy groups was significantly higher than that in the control group (*P* < 0.05) (Figure 3(a), Table 2.2). (2) The expression rate of CD4^+^ in each group was as follows: control group 21.05 ± 13.32 and ISE group 27.15 ± 15.48, no statistical difference (*P* < 0.05) (Figure 3(b), Table 2.2).

The expression of PD-1 in CSF of patients with IE was upregulated in CD4^+^CD25^high^ Treg cells, and IL-10 increased simultaneously. (1) The expression rate of PD-1+CD4^+^CD25^high^ Treg in each group was as follows: control group 19.37 ± 4.51 and ISE group 50.45 ± 29.56; the ISE group was significantly higher than the control group (*P* < 0.05) (Figure 4(a), Table 2.2). (2) There was no significant difference in the ratio of PD-1+CD4^+^CD25^high^ Treg/CD4^+^CD25^high^ Treg in two groups: *Z* = 1.645 (*P* > 0.05) (Figure 4(b)). (3) The correlation coefficients of the ISE group were as follows: PD-1+CD4^+^CD25^high^ Treg (-0.391), PD-1+CD4^+^CD25^low^ Treg (0.447^∗^), CD4+CD25^low^ (0.109), CD4^+^CD25^high^ (0.378), IL-10 (0.205), P1 (-0.318), P2 (0.204), in which age is related to PD-1+CD4^+^CD25^low^, upregulated with age (*P* < 0.05). Gender, attack frequency, and course are not related factors affecting central immune regulation (Figure 4(c)). (4) The concentration of IL-10 in CSF was as follows: control group 4.78 ± 1.63 pg/ml and ISE group 66.68 ± 15.56 pg/ml. The patients in the ISE group were significantly higher than those in the control group (*P* < 0.05) (Figure 4(d), Table 2.2). (5) The concentration of IL-6 in CSF was as follows: control group 1.89 ± 1.84 pg/ml and ISE group 2.59 ± 1.76 pg/ml; there was no significant difference (*P* > 0.05) (Figure 4(e), Table 2.2).

The article "PD-1 Is an Immune-Inflammatory Potential Biomarker in Cerebrospinal Fluid and Serum of Intractable Epilepsy" was retracted in 2024. Reasons: signs of a paper mill; compromised peer review; unreliable results or conclusions.

## 4. Discussion

In this study, we first assessed PD-1 levels in CSF and serum samples from patients with IE. We found lymphocyte ratio was decreased and PD-1+CD4^+^CD25^high^ Treg level was increased in the patients with IE, compared with controls (Figure 4(a), Table 2.2). Interestingly, PD-1 levels were not affected by AEDs and treatment course, but by epilepsy onset level (Tables 1.1 and 2.1). These results supported that PD-1 might be involved in the pathogenesis of IE. At the same time, we also found mild inflammation in patients with IE; both IL-6 and IL-10 were increased in serum samples (Figures 2(d) and 2(e), Table 1.2). The upregulation rate of IL-10 was more significant than that of IL-6. But in CSF, the upregulation of IL-10 was the main expression (Figure 4(d), Table 1.2), which was consistent with the immune effect caused by overexpression of PD-1 in CD4^+^CD25^high^ Treg cells. The expression of PD-1 in CD4^+^CD25^high^ Treg cells of the group with PS was also positively correlated with age but not about gender, which was consistent with the previous study of Vieira et al. [19]. These results indicated that age was a related factor of immune regulation. Thus, we suspected that the decreased immune response of lymphocytes of patients with IE was due to the decrease of absolute number and/or ratio of lymphocytes. The increased expression of PD-1 in CD4^+^CD25^high^ Treg cells promoted the inhibitory function of Treg cells, reduced T cell proliferation, inhibited effector T cell activation, which led to the decline of immune response finally. We also found that the increase of IL-10 expression was the main trend of inflammatory factors, which was consistent with the expression trend of PD-1+CD4^+^CD25^high^ Treg cells. It was indicated that the increase of IL-10 reduced APC antigen-presenting ability. It blocked proliferation of T cells activated by antigen and secretion of other inflammatory mediators and decreased the activity of T cells and the ability of immune response indirectly. The anti-inflammatory ability was closely related to age but not with gender (increased with age).

The article "PD-1 Is an Immune-Inflammatory Potential Biomarker in Cerebrospinal Fluid and Serum of Intractable Epilepsy" was retracted in 2024. Reasons: signs of a paper mill; compromised peer review; unreliable results or conclusions.

The inhibitory receptor PD-1 is a member of the CD28/B7 family and is inducibly expressed on T cells, natural killer T cells (NKT), B cells, monocytes, and dendritic cells (DCs). Those mainly regulate the lymphocyte function in the activated state [20]. PD-1 interacts with its ligands PD-L1 and PD-L2 [14]. PD-L1 is constitutively expressed on hematopoietic and nonhematopoietic cells and in immunoprivileged sites (eye, placenta) and is highly expressed in inflammatory environments. Upon general activation of the immune response, professional antigen-presenting cells (APCs) and T cells further augment their PD-L1 expressions. By contrast, PD-L2 is inducibly expressed only on macrophages, DCs, and bone marrow-derived cultured mast cells. PD-1 is the only inhibitory receptor of the coinhibitory molecules whose ligands are expressed both in lymphoid and nonlymphoid organs [14]. This might explain why the PD-1-PD-L1 pathway has been postulated to regulate immune responses both in lymphoid and nonlymphoid organs including the brain. Therefore, PD-1 plays a vital role in the maintenance of peripheral and central tolerance (i.e., mechanisms that maintain the quiescence of autoreactive T cells that have already matured and escaped the mechanisms of central tolerance during development in the thymus). CD4^+^CD25^high^ Treg cell is a kind of T cell subgroup that plays an important role in inhibiting the proliferation in autoimmune response and maintaining the immune stability. It mediates immune tolerance by producing inhibitory cytokines [21]. When CD4^+^CD25^high^ Tregs decrease, the inhibition function is damaged, and the surface molecule expression is defective, which can cause the occurrence and development of autoimmune diseases [22]. To study on the immune pathway of PD-1 negative regulation, we need to start with the number and ratio of its expression in CD4^+^CD25^high^ Treg cells. The experimental model of peripheral immune disease supports the role of PD-1-PD-L on Treg cells, and it is found that PD-1+CD4^+^CD25^−^ T cell subgroups can inhibit the progress of peripheral immune disease [23].

A line of evidence suggests that the PD-1–PD-L pathway plays a central role for the dysfunction of T cell and chronic infection in central nervous system diseases. Saresellaa et al. [24] found that PD-1^neg^ Treg cells might play an important role in the pathogenesis of Alzheimer's disease; loss of such cells and their functional ability is associated with development of Alzheimer's disease by studying the expression of PD-1 in different subgroups of Treg cells in patients with cognitive impairment and Alzheimer's disease. Ishizaki et al. [25] found that PD-1 gene contributed to a genetic susceptibility to subacute sclerosing panencephalitis (SSPE) by investigating a functional difference in promoter activity of two haplotypes and compared the expression levels of PD-1 between SSPE and controls. There are innate immune activity and acquired adaptive immunity in the process of epilepsy [26]. Both of them can produce pathogenicity to the brain through immune reaction. In chronic disease stage, the PD-1 pathway normally gets activated and is involved in promoting tolerance and preventing tissue damage. In our study, the increased expression of PD-1 on CD4^+^CD25^high^ Treg cells and the decreased expression of the lymphocyte in IE patients indicate that Tregs can be exhausted and their capability of suppression can be compromised. We observed that IL-6 in peripheral blood of patients with IE was increased, but there was no significant difference in CSF, similar to previous studies [27]. The IL-6 level in plasma did not reliably reflect its brain level. It was considered that the changes might be related to the seizure closely for the stress response and the excitability of neurons. Previous studies found that the concentrations of IL-6 were fluctuated according to the types and treatment stages of epilepsy [28, 29]. Previous results showed the significant rise of IL-6 in plasma after seizures both in TLE without hippocampal sclerosis (HS) [30] and in TLE group [31]. It remains unclear whether elevated blood levels of IL-6 allow a conclusion to be drawn about its expression and function in epileptogenic brain areas. Therefore, it is necessary to explore the role of IL-6 in epilepsy. IL-10 is the main cytokine of Tregs to exert their inhibitory actions. Several animal studies and clinical observations suggest that IL-10 has anticonvulsant effect and has protective effect on epileptiform activity induced by transient hypoxia in rat hippocampal slices [32, 33]. Importantly, IL-10 promotes the production of TGF-*β* and controls the response of target cells to TGF-*β*. TGF-*β* produced by iTregs can induce other immature CD4^+^CD25^low^ cells to become similar inhibitory cells. We observed that IL-10 secreted by Tregs from IE patients (Figures 2(d) and 4(d)) was more than that from the control, which shows the immunosuppressive effect. Whether it is the protective effect or the triggering factor for epilepsy, we need further study.

The article "PD-1 Is an Immune-Inflammatory Potential Biomarker in Cerebrospinal Fluid and Serum of Intractable Epilepsy" was retracted in 2024. Reasons: signs of a paper mill; compromised peer review; unreliable results or conclusions.

Some limitations of this study should be mentioned. First, this study only had investigated PD-1 expression in IE patients; we did not assess the mechanism research. Second, the patients of the PS group are outpatients, so CSF has not been obtained again for this study. Third, PD-1 levels were not determined in a large sample size because of difficulties in obtaining CSF samples from IE patients and controls. Fourth, we should measure some of oxidative stress parameters and some other inflammatory cytokines in serum or CSF. Fifth, we did not analyze the effect of seizure control on PD-1 levels because many patients were uncertain about their baseline seizure frequency.

## 5. Conclusion

Overall, our study indicates higher CSF- and serum-PD-1 levels in IE patients. Therefore, CSF- and serum-PD-1 amounts should be considered candidate biological markers in intractable epilepsy. However, these findings require further confirmation. Studies with larger sample size, regular follow-up, and therapeutic effect would enable a comprehensive assessment of the potential role of PD-1 in intractable epilepsy.

## Figures and Tables

**Figure 1:** (a) The positive rate of peripheral blood lymphocytes. The PS group and the ISE group were significantly lower than the control group, and the ISE group was significantly lower than the PS group. (b) The rate of CD4^+^ T lymphocyte expression in peripheral blood. The PS group and the ISE group were significantly lower than the control group. The ISE group was significantly lower than the PS group.

**Figure 2:** (a) The expression level of PD-1 expression on CD4^+^CD25^high^ Treg lymphocytes of two groups. Patients with intractable epilepsy were significantly higher than the control, and the expression level of the ISE group was significantly higher than that of the PS group. (b) The patients with IE were significantly higher than the control group; the ratio increased with the degree of seizure increased. (c) In the PS group, the relationship between the age of PD-1+CD4^+^CD25^low^ T cells and the percentage of CD4^+^ T cells (P2) was correlated with the age in peripheral blood. Age increased and expression decreased. (d) IL-10 levels in the PS group and the ISE group were significantly higher than those in the control group, and the ISE group was significantly higher than the PS group. (e) IL-6 levels in the PS group and the ISE group were significantly higher than those in the control group, but there was no significant difference between the ISE group and the PS group.

**Figure 3:** (a) The expression rate of lymphocytes in the cerebrospinal fluid of patients with ISE was significantly higher. (b) The positive rate of CD4^+^ T lymphocytes in the control group and the ISE group has no significant difference.

**Figure 4:** (a) Expression of PD-1 on CD4^+^CD25^low^ and CD4^+^CD25^high^ Treg lymphocytes in cerebrospinal fluid in patients with ISE. (b) The rate of PD-1+CD4^+^CD25^high^ Treg/CD4^+^CD25^high^ Treg. (c) Age correlates with PD-1+CD4^+^CD25^low^ (Table 2.4). (d) The level of IL-10 in cerebrospinal fluid. (e) The level of IL-6 in cerebrospinal fluid.

The article "PD-1 Is an Immune-Inflammatory Potential Biomarker in Cerebrospinal Fluid and Serum of Intractable Epilepsy" was retracted in 2024. Reasons: signs of a paper mill; compromised peer review; unreliable results or conclusions.

**Table 1:** Comparison of clinical features of patients and controls.

	Control (*n* = 25)	PS (*n* = 41)	ISE (*n* = 26)	*P* value
Gender: male (refer to female)	40.00%	48.78%	45.83%	0.785^a^
Age (years)	31.8 ± 7.21	28.1 ± 6.19	27.85 ± 3.61	0.065^b^
Course of disease (days)	—	9.15 ± 5.77	8.60 ± 3.67	0.752^b^

Note: ^a^chi-square test, double tail; ^b^Kruskal-Wallis rank sum test.

## Data Availability

Data in this research were uploaded as the supplemental files. All data generated or analyzed during this study are included in this article.

## Supplementary Materials

Supplementary Materials (1) Data in peripheral blood of the experimental groups and the control group. Table 1.1: comparison of clinical features of patients and control. Table 1.2: the expression of PD-1 and IL-10/IL-6 in peripheral blood of the experimental groups and the control group. Table 1.3: comparison of CD4+CD25high+PD-1+Treg/CD4+CD25high Treg ratios between experimental and control groups. Table 1.4: age correlates with each outcome in the PS group. Table 1.5: age correlates with each outcome in the ISE group. (2) Data in cerebrospinal fluid of the experimental groups and the control group. Table 2.1: comparison of clinical features of patients and control. Table 2.2: the expression of PD-1 and IL-10/IL-6 in cerebrospinal fluid of the experimental group and the control group. Table 2.3: age correlates with each outcome in cerebrospinal fluid of the ISE group.
